The article "The Outcome of Artisan Intraocular Lens Implantation in Children: A Narrative Review" was published in 2024. Journal: Cureus.

# The Outcome of Artisan Intraocular Lens Implantation in Children: A Narrative Review

**DOI:** 10.7759/cureus.59435

**Published:** 2024-05-01

**Authors:** Mitra Akbari

**Affiliations:** 1 Department of Eye, Eye Research Center, Amiralmomenin Hospital, School of Medicine, Guilan University of Medical Sciences, Rasht, IRN

**Keywords:** intraocular lens, iris claw, capsular support, pediatric aphakia, artisan lens

## Abstract

Aphakia is a condition in which the eye's crystalline lens is not in its proper position because of a perforating injury, surgical removal, dislocation of the lens, or congenital anomaly. The management of aphakia can be either conservative or surgical. Various surgical techniques could be used, including retro pupillary-fixated iris-claw intraocular lenses (IOLs) and anterior-fixated iris-claw IOLs. One of the challenges faced by ophthalmologists is the optical rehabilitation of pediatric aphakic patients because a child's eye is still growing, resulting in fundamental variations in their refractive elements, and the immature visual system faces the risks of amblyopia development in the case of defocus or inequality of visual input between both eyes. There is also the risk of the incidence of side effects that can be accepted in adults but not in children. Finally, accurate postoperative supervision and optical rehabilitation in pediatrics will be more complex than that in adults. This review showed that it is possible to place, replace, and exchange the Artisan IOL with minor surgical trauma. Hence, this procedure can be an acceptable therapeutic method for correcting the developmental refractive changes of the growing aphakic eye. However, some worries are still caused by probable long-term side effects, including endothelial cell loss. Finally, a significant attempt at visual rehabilitation is to treat pediatric aphakia with Artisan IOL.

## Introduction and background

Aphakia is a condition where a congenital anomaly, surgical excision, dislocation, or perforating injury malpositions the crystalline lens of the eye [1]. This condition is characterized by the absence of the natural lens of the eye, which typically occurs subsequent to cataract surgery. Extraction of the lens disrupts the equilibrium of intraocular fluids and structures. For example, in the absence of a lens, the vitreous humor (a gel-like substance) and the anterior segment (the front portion of the eye) experience compositional and pressure variations. Impaired vision could lead to complications like elevated intraocular pressure (IOP) or retinal detachment [2]. Loss of accommodation, high hyperopia, and anisometropia are some of the consequences [3].

Various surgical techniques, such as transscleral fixation with sutures, intrascleral fixation without sutures, iris-sutured intraocular lenses (IOLs), retropupillary-fixated iris-claw IOLs, and anterior-fixated iris-claw IOLs, can correct aphakia [4]. One of the hardest things for ophthalmologists is helping pediatric aphakic patients with optical rehabilitation because a child's eye is still growing, so the refractive elements are changing in fundamental ways. Also, the visual system is still developing, so defocus or unequal visual input between both eyes can cause amblyopia. There is also the risk of side effects that can be accepted in adults but not in children. Finally, accurate postoperative supervision and optical rehabilitation in pediatrics will be more complex than in adults [5-8].

Children with aphakia could benefit from a variety of surgical alternatives. Experts in the field suggested various surgical approaches and IOL plans, such as the implantation of the Artisan aphakia IOL, with their specific merits and demerits [4]. During a surgical procedure, a surgeon inflates the Artisan IOL to the iris. Recently, researchers have also implanted Artisan IOLs retropupillarily [9]. Studies in the past have shown that this lens can be successfully implanted in children with myopic anisometropic amblyopia, congenital cataracts, traumatic cataracts, and other conditions [10,11]. However, surgical corrections for children with aphakia who do not have adequate capsular support imply a challenging route traveled by the ophthalmic surgeons [4], and inadequate research has been performed on the secondary results of IOL implantation’s long-term vision, especially about Artisan IOL.

A review of the literature on surgical management of pediatric aphakia when there is insufficient capsular support examined the pros and cons of the available techniques. The study revealed that the placement of anterior Artisan IOLs is more straightforward than other methods. However, more research is necessary to determine the long-term effects of these techniques on corneal endothelial cell loss (ECL) [4].

Overall, IOL implantation in the cases of pediatric eyes with aphakia is a difficult task yet, but surgeons have numerous IOL alternatives to treat. Therefore, this research aimed to review papers evaluating the consequences of Artisan IOL implantation, a relatively new technique, in children with aphakia, considered a high-risk group.

## Review

Method

Inclusion and Exclusion Criteria of Review

Using the research databases Web of Science, EMBASE, and PubMed, we identified the papers related to the Artisan aphakic IOL from November 1, 1986 (when the first implantation took place) until December 31, 2022. Hence, we have selected the following keywords: "paediatric" or "children" and "aphakia" and "Artisan lens" or "Artisan aphakia IOL" or "Iris-claw Artisan IOL" or "iris-claw IOL" or "Iris-claw intraocular lens." The review included all relevant case reports, case series, and human clinical trials but excluded reviews and non-English research. The selected publications provided additional information, such as the year of publication, first author(s), research design, sample size, and critical results.

Results

The study included 32 articles, including case reports and clinical trials. Table 1 presents the main results of the studies.

**Table 1:** Publications presented on Artisan IOL in pediatric aphakic patients. BCVA: best-corrected visual acuity; IOL: intraocular lens; ECL: endothelial cell loss; VA: visual acuity; RPIC-IOL: retropupillary iris-claw intraocular lens, ECC: endothelial cell count; SFIOL: scleral-fixated intraocular lens; CDVA: corrected distance visual acuity; UDVA: uncorrected distance visual acuity; IOP: intraocular pressure; D: diopter; PCIOL: posterior chamber intraocular lens; ICIOL: iris-claw intraocular lens; IFIOL: iris-fixated intraocular lens.

Study (author and year)	Study design	Sample size N (%)	Summary of results
Van der Pol et al. (1996) [12]	Prospective investigation of ICIOL in children	27 (38%)	ICIOL was a very adaptable IOL, and it is possible to use it in numerous cataract procedures. It is possible to remove and exchange it with minor surgical trauma. Visual acuities outcome could be compared to the consequences in other series
Chipont et al. (2001) [13]	Case report of anisometropic amblyopia with spherical equivalent refraction	1 (2%)	VA six months following the surgical operation was 20/25 in one eye and 20/20 in another eye, but its stability was observed after 18 months of surgical operation
Saxena et al.(2003) [14]	Prospective case report of anterior chamber IFIOL for anisometropic amblyopia	1 (1%)	The BCVA was 1 after one year, and it remained stable through three years. Binocular stereovision developed. Although postoperative ECL was significant, there were no complications
Lifshitz et al.(2004) [15]	Retrospective study of Artisan IOL for idiopathic subluxated lenses	3 (4%)	Postoperative BCVA 6/12 or more in three patients. VA improvement by two or more Snellen lines in each eye. There were no side effects
Neuhann et al. (2005) [16]	Case report of an IFIOL in a 3-year-old child following a perforating injury	1 (1%)	Considerable formation of non-inflammatory fibrous membrane in the anterior chamber that involves the present IFIOL with need for explantation. A retrocorneal membrane was caused by corneal stroma that created a "cocoon" membrane on the ICIOL
Lifshitz et al. (2005) [17]	Case report of unilateral cataract extraction and PCIOL implantation	1 (1%)	A residual progressive myopic error after the first surgery. After 9 months of the second operation, myopia diminished. No complications were observed after the secondary implantation of Artisan
Aspiotis et al. (2006)[18]	Retrospective study of children with subluxated lenses caused by Marfan syndrome	5 (7%)	VA improvement by ≥4 Snellen lines in each eye. ECC was fixed in each case at a six-month follow-up interval. No complications during surgery
Odenthal et al. (2006) [19]	Examination of retrospective ECL following the Artisan IOL for congenital and traumatic cataract	10 (10%)	ECL was 41% in the traumatic cataract group. Any statistical differences in ECC between operated and unoperated eyes in the congenital cataract group. There was a relationship between ECL with original corneal scar length of the trauma
Sminia et al.(2008) [20]	Retrospective evaluation of Artisan IOL for aphakia after trauma	5 (5%)	Mean ECL was 40%. Postoperative BCVA equaled 20/40 or better in four eyes. Complication included retinal detachment 19 months following the primary injury event in one eye
Sminia et al.(2011) [21]	Retrospective investigation of the Artisan IOL in children with aphakia and partial aniridia because of trauma.	5 (5%)	VA improved and showed stability in both eyes but diminished in one eye. An acceptable cosmetic result was found in three patients. Mean spherical equivalent refraction error was −4.0 D at the end of the follow-up session. Mean ECL was 42%. Complications: persistent anterior uveitis, partial luxation of the IOL, secondary glaucoma, and retinal detachment
Sminia et al. (2011) [21]	Retrospective assessment of ECL after Artisan IOL for congenital and traumatic and cataract	10 (20%)	Postoperative mean ECC that could be compared to the mean normal ECC for the respective cases
Sminia et al. (2012) [22]	Retrospective evaluation of Artisan IOL for ectopia lentis in Marfan syndrome	2 (4%)	Acceptable postoperative visual outcomes. Without chronic IOL-related side effects. ECC in the estimated range for normal eyes
Cleary et al.(2012) [23]	Retrospective evaluation of Artisan ICIOL for ectopia lentis	5 (8%)	Mean postoperative ECL was 14.2% (P<0.001). Postoperative mean VA was 0.04±0.09 logMAR. No complications were observed
Siddiqui and Khan (2013) [24]	Prospective investigation of visual results and ECC following the Artisan IOL for lens subluxation	11 (18%)	Mean postoperative ECL: 17.1%. Mean postoperative BCVA: 0.26±0.13 logMAR (P=0.001)
Zafar et al. (2013) [25]	Prospective evaluation of central corneal thickness and intra ocular pressure in eyes suffering from the crystalline subluxated lenses after Artisan IOL fixation	17 (17%)	Mean pre/postoperative IOP: Group A (primary Artisan IOL) 14.88 and 14.16/Group B (secondary Artisan IOL) 12.44 and 14.44. Mean pre/postoperative central corneal thickness: Group A 529.13 and 529.87/Group B 567.33 and 568.83
Gonnermann et al. (2013) [26]	Retrospective cohort study of posterior iris-claw aphakic IOL	4 (7%)	Preoperative VA: 0.60 logMAR/postoperative VA: 0.13 logMAR (statistically significant difference). Mean postoperative ECL: 6.4%. Complications: transient postoperative hypotony and traumatic dislocation of IOL
Xue et al. (2013) [27]	Prospective evaluation of retropupillary Artisan in aphakia following penetrating eye injuries	3 (3%)	The patients achieved BCVA of 20/25 to 20/30 at 8, 13, and 22 months of follow-up
Gawdat et al. (2015) [28]	Prospective consequences of Artisan IOL for aphakia	18 (25%)	Postoperative BCVA for lens subluxation and traumatic aphakia ameliorated to 0.3±0.2 logMAR (P<0.001) and 0.38±0.15 logMAR (P<0.002). Significant decrease of ECC, one year after surgery (2892.64±441.79 cells/mm^2^). Side effects: pupillary block (n=1) and traumatic dislocation (n=2)
Brandner et al. (2015) [29]	Retrospective study of RPIC-IOL for Aphakic Eyes	10 (15%)	Median VA improved by 0.12 logMAR. Mean postoperative spherical equivalent was determined to be -0.05±1.76 D. Any chronic side effects, only a haptic disenclavation with IOL subluxation instantly following an automobile accident in one patient
Kavitha et al. (2016) [30]	Retrospective outcomes of Artisan IOL vs. PCIOL for traumatic cataract	50 (50%)	1) BCVA outperformance in each group. Any significant differences were not observed in BCVA logMAR between groups. Side effects in the Artisan IOL group: cystoid macular edema (n=1), secondary glaucoma (n=1), and IOL de-enclavation (n = 1)
Hildebrand et al. (2016) [31]	Prospective evaluation of RPIC-IOL for congenital, developmental cataract or penetrating eye injury	8 (8%)	Three eyes with penetrating injury and one with developmental cataract; however, any pre-existing amblyopia did not achieve final BCVA 0.00-0.10 logMAR. Four eyes with pre-existing dense amblyopia caused by permanent unilateral cataract reached final BCVA 0.50-1.00 logMAR. Final spherical equivalent -2.02 D ±0.87:1.78 D±0.84 myopic shifted from the target SE. Complications: transient postoperative uveitis (n=2) and accidental IOL dislocation caused by blunt trauma (n=1)
Manning et al. (2016) [32]	Retrospective results following the Artisan IOL implantation for ectopia lentis in Marfan syndrome	8 (16%)	Mean postoperative ECL: 15.4%. Mean postoperative BCVA: 0.12±0.19 logMAR. Complications: de-enclavation (n=1) and pupillary block (n=1)
Catala-Mora et al. (2017) [33]	Prospective evaluation of Artisan IOL for ectopia lentis	12 (21%)	1) Mean BCVA improvement from 0.91±0.29 logMAR to 0.18±0.23 logMAR. Postoperative ECL: 5.04%±9.58%. Annual ECL rate: 3.16%±4.46%. Complications: cystoid macular edema (n=1), retinal detachment (n=1), and traumatic IOL dislocation
Çevik et al. (2017) [34]	Retrospective evaluation of ICIOL implantation in patients suffering from non-traumatic ectopia lentis.	17 (30%)	BCVA values were increased. Target refraction values were achieved 47% in group with hereditary disease and 22% in group without hereditary disease. The presence of post-surgery lens dislocation and hypotonia in both groups, but retinal detachments were observed in three patients from group with hereditary disease
Wasik et al.(2018) [35]	Electron microscopic evaluation of an explanted retropupillary Artisan lens	1 (1%)	No biofilm or cellular deposition on the RPIC-IOL surface was significant three years after implantation
Rastogi et al. (2018) [36]	Prospective assessment of primary RPIC-IOL in cases suffering from large lens subluxations	14%	BCVA increase with the mean 0.351±0.154 logMAR units in comparison with the preoperative value of 0.771±0.132 logMAR units (P=0.003). Mean ECC decreased by 0.99%. The lens position was parallel to the iris plane in each at the end of a six-month follow-up interval
Shuaib et al. (2019) [37]	Prospective randomized clinical study of transscleral sutureless IOL versus RPIC-IOL fixation for paediatric aphakia	30 (30%)	Improvement in BCVA without any differences between the groups. ECC was reduced in the two groups without any significant differences between groups. Side effects: transscleral-fixated IOL group: ocular hypertension and IOL decentration, ICIOL group: glaucoma, haptic disenclavation, and retinal detachment
Muthukumar et al. (2022) [38]	Retrospective comparisons of retropupillary-fixated iris claw lens vs. sclera-fixated lens in the children with aphakia secondary to ectopia lentis	38 (57%)	Mean BCVA improved (logMAR) in both groups (retropupillary IFIOL: from 1.5±0.2 to 0.3±0.2, SFIOL: from 1.5±0.3 to 0.3±0.2). No serious complications in either of the groups
Rastogi et al. (2022) [39]	Prospective evaluation of RPIC lens versus Gore-Tex assisted SFIOL in children with large lens subluxations	60	BCVA improvement in RPIC-IOL group: 0.28±0.41, in SFIOL group: 0.44±0.45 logMAR. Significant IOL tilt in four eyes in RPIC-IOL group and five eyes in SFIOL group. Astigmatism mean change 4.38±5.9D in RPIC-IOL group and 4.91±4D in SFIOL group. No significant posterior segment complications were seen
Fuerst et al. (2014) [40]	Prospective analysis of implantation of Artisan aphakia IOL for non-traumatic ectopia lentis in children.	28 (56%)	Mean BCVA improvement from 0.36 to 0.18 logMAR. Five reoperations were needed, three related to post-implantation trauma. Mean increase in central corneal thickness was 11.9 μm higher postoperatively. Mean loss of corneal ECC postoperatively was not significantly different from 0
Griščíková et al. (2021) [41]	Anterior chamber IFIOL implantation for treatment of high anisometropia	71 (71%)	UDVA improved from 1.74±0.36 to 0.45±0.28 logMAR. The mean CDVA altered from 0.68±0.32 to 0.27±0.15 logMAR. The mean preoperative ECC of 2874.7 shifted to 2685.3 cells/mm^2^. No serious complications or loss of Snellen lines of CDVA

In 1996, an iris-fixated one-piece iris-claw IOL (ICIOL) was employed to treat 27 children with cataracts. The study demonstrated the versatility of the lens, enabling its application in various cataract procedures and its removal and exchange with minor surgical trauma [12]. A boy who was 8 years old had myopic anisometropic amblyopia. In 2001, doctors decided to treat him with an Artisan iris-claw phakic anterior chamber IOL and occlusion therapy, which reversed the amblyopia [13].

Moreover, occlusion therapy for additional treatment of the amblyopic eye was followed in a child with the iris-fixated Artisan phakic IOL implantation in 2003 for supporting the anisometropic amblyopia therapy and correcting high unilateral myopia; however, the best-corrected visual acuity (BCVA) was 1 in the amblyopic eye one-year post-operation, and development in binocular stereovision was observed. Furthermore, despite significant postoperative ECL, a three-year follow-up revealed stable visual acuity (VA) and no side effects [14]. In addition, BCVA was 6/12 or better in three cases after surgery in a case series of four eyes suffering from idiopathic subluxated lenses. The tests showed that each eye's VA improved by two or more Snellen lines, and each eye's postoperative spherical equivalent ranged from ±1.00 diopter. There were no significant side effects [15].

According to a study of a three-year-old child who underwent repairing a corneal injury, Artisan IOL implantation, as well as crystalline lens extraction following a penetrating injury in 2005, histopathologic analyses showed compatibility with a retro corneal membrane caused by the corneal stroma, forming a "cocoon" membrane on the ICIOL [16]. In another examination, experts in the field conducted posterior chamber intraocular lens (PCIOL) implantation and unilateral cataract extraction on one of the eight-week-old infants. They showed a residual progressive myopic error after six months and at the age of three years. Then, they performed secondary implantation of the Artisan phakic IOL. They found no side effects, but myopia declined nine months after the subsequent surgery. The 2005 study demonstrated that Artisan IOL implantation is among the most straightforward methods, observing the major ECL during surgical procedures without significant cell losses [17].

In 2006, a case series of seven eyes with subluxated lenses due to Marfan syndrome underwent lens extraction and Artisan implantation without any complications. Each eye showed a VA improvement of approximately four Snellen lines, and the endothelial cell status remained constant in a six-month follow-up [18]. In 2006, another study discovered that 10.5 years after implanting an iris-fixated intraocular lens (IFIOL) to treat traumatic cataracts, ECL was still excellent because of the link between the length of the corneal scar and the injury. Researchers found no differences in the endothelial cell density between the operated and unoperated eyes of children with congenital cataracts [19].

In 2007, research demonstrated that Artisan aphakia IOL implantation could serve as a therapeutic option for children with aphakia who lack capsular support due to trauma [10]. According to the results of one study in 2008, the Artisan IOL is one of the therapeutic options for aphakia as a result of penetrating ocular trauma in the respective children. Furthermore, researchers should focus on the high-risk features of the treated eyes and the significance of accurate patient selection in the surgery’s outcomes [20]. In 2011, a cohort of children undergoing juvenile cataract removal or bilateral congenital disabilities with Artisan implants exhibited an average count of 2702 endothelial cells per square millimeter (ECD), which is comparable to the average count of normal endothelial cells (ECC) [21].

A study in 2012 [22] found that in two patients suffering from bilateral crystalline lens dislocation and Marfan syndrome who underwent Artisan implantation and lens extraction, one of the acceptable visual outcomes was the absence of an acute side effect and ECDs in the estimated ranges for eyes without cataract surgery. Another study in 2012 showed that Artisan implants were safe and efficient in correcting children’s aphakia after lensectomy for ectopia lentis, which empowered them to have appropriate spectacle-free distance vision in 75% of eyes without any postoperative consequences [23].

Research from 2013 demonstrated that Artisan IOL is a safe surgical option for managing ectopia lentis in children, with minimal side effects and less eye trauma [24]. A 2013 study revealed that primary and secondary Artisan IOL did not significantly alter corneal thickness or IOP during the follow-up period [25]. One more study in 2013 [26] accompanied the posterior implantation technique of Artisan IOL with satisfactory visual results and acceptable rates of complications. Another study in 2013 presented three children with a penetrating eye injury that led to aphakia but experienced successful repair by retropupillary Artisan IOL. Finally, the children exhibited BCVAs of 20/25 to 20/30 at follow-up [27].

In a 2015 study, the mean preoperative logMAR BCVA was 0.95 for traumatic patients and 0.7 for patients with subluxation, which improved to 0.38 and 0.3 in the postoperative one-year follow-up. The one-year follow-up showed a reduction in the central ECD. The analyses revealed the development of traumatic dislocation and pupillary block in two cases and one case, respectively. Overall, Artisan IOL implantation for pediatric aphakia has demonstrated an acceptable level of visual outcome [28]. Another study in 2015 revealed that Artisan IOL implantation behind the iris was not harmful to children without capsular support and yielded excellent visual outcomes with lower rates of complications [29].

One study from 2016 showed that both iris-fixed (IFIOL) and posterior chamber (PCIOL) implantations would improve the vision of children with traumatic cataracts with no significant side effects after surgery [30]. In these situations, we could use IFIOL instead of PCIOL. In 2016, another study added more support for the retropupillary Artisan IOL in young children who had trouble getting their lenses taken out because of developmental or congenital cataracts and injuries that went through the eye [31]. In 2016, a cohort study examined children with ectopia lentis and Marfan syndrome with one or more intraocular procedures. The study found that the rate of retinal detachment did not rise, which led to a moderate rate of ECL [32].

According to a prospective cohort study (2017) of 21 eyes who suffered from chronic ectopia lentis with VA <20/63 and thus experienced lensectomy, vitrectomy, anterior chamber Artisan implantation with iris-claw elevation using pars plana, as well as iridectomy, this technique is feasible, and lifespan ophthalmic follow-up, such as central ECC measurement, fundus examination, and IOL position monitoring, must be implemented in such cases [33]. In 2017, a study categorized 70 children with nontraumatic ectopia lentis into groups with and without hereditary disease and found that their BCVA values improved following the surgical operation. Researchers have also observed lens dislocation and hypotonia. Additionally, they have noted retinal detachments in three patients from a hereditary disease group [34].

In 2018, an electron microscope study of an explanted retropupillary Artisan lens that had been implanted three years before showed that the surface of the retropupillary iris-claw intraocular lens (RPIC-IOL) did not have any biofilm or cellular deposition. In particular, it is considerable in cataract surgeries in younger children with the highest risk of amblyogenic opacification of the visual axis [35]. In 2018, 14 eyes suffering from lens subluxations underwent a basic procedure known as pars plana lensectomy-vitrectomy, including placing an ICIOL in the retropupillary position. Postoperative examination showed increased BCVA in each patient. The lens position has also been parallel to the iris plane in each case at the end of the six-month follow-up. According to this study, children with large lens subluxations can think about primary implantation of RPIC-IOL as one of the best and safest options, similar to scleral-fixated PCIOLs in some ways [36].

Shuaib’s study in 2019 showed that RPIC-IOL lens fixation has been proposed as one of the shorter procedures that is technically simpler than sutureless transscleral fixation; however, disinclination risk must be mainly addressed in children. Therefore, people consider scleral fixation the only alternative for chronic iris damage, but it has a higher correlation with ECL [37].

Examining the kids who had lens subluxation because of ectopia lentis and had scleral-fixated intraocular lens (SFIOL) implanted or retropupillary iris-fixated IOLs in 2021 showed that their eyes did not have any severe problems. IOL scleral fixation or retropupillary iris would be a safe and effective way to fix ectopia lentis [38].

A 2022 study on the RPIC-IOL and SFIOL in children with big lens subluxations revealed no significant posterior segment issues with either technique. Both procedures had comparable visual outcomes. Patients with a high risk of retinal detachment may prefer RPIC-IOL implantation due to its speed and ease of use [39]. Another study reported the long-term consequences of iris-claw aphakia IOL implantation for nontraumatic ectopia lentis in children. The IOL exhibited a perfect safety profile in the children [40]. In 2022, another study found that an iris-fixated phakic IOL is one of the safest and most effective ways to treat nearsightedness, farsightedness, and high anisometropic myopia in kids who cannot wear glasses or contacts [41].

Discussion

Early diagnosis and appropriate clinical care can lead to the best outcomes for pediatric aphakia. Congenital cataracts are one of the most important reasons children have aphakia, which has characteristics such as vision loss and amblyopia. It is also one of the treatable causes of vision loss in childhood [42]. The necessity for cataract treatment is different according to cataract progression as well as the density of opacities at birth and in the course of childhood [43]. The management of aphakia can be either conservative or surgical. Spectacles or contact lenses are the conservative treatments [44]. 

As mentioned earlier, aphakia correction with aphakic glasses has been explained without parents’ collaboration or in infrequent cases [5]. The literature also provides limited evidence about contact lens correction for pediatric aphakia [45]. It seems that surgical management of children's aphakia is the best way. However, pediatric cataract surgeons advocate for primary IOL implantation in cases older than two years, a practice still controversial for younger children due to the higher risk of postoperative complications [46]. Postoperative intraocular inflammation is usually more severe in younger children. Additionally, in cases under two years old, lens implantation following cataract removal may cause a myopic shift [43,47,48].

With sufficient surgical experience and rigorous follow-up, IOL implantation may have an acceptable complication rate in children up to 2 years old with bilateral cataracts [46]. We must make careful decisions about the implantation lens schedule for children, considering factors such as the patient's age, potential consequences, the cost-effectiveness of the treatment for their families, and the selection of the appropriate IOL type and power [43]. Research demonstrates that when an experienced surgeon performs elective surgery after elementary school age, the risk of high myopia and complication rate is low, the predictable refractive outcome is higher, and there are fewer adverse events [49].

Research has shown that developing countries have a lower complication rate for IOL implantation in children. Patient selection criteria, age at the onset of the surgical operation, type, place of study, and postoperative care would be potential reasons [50]. Various countries continue to see alterations in managing patients with aphakia, and a fixed referral clinical network is crucial to achieving desirable outcomes.

The most recent study (2022) regarding the outcome of Artisan IOL implantation in children with aphakia was a large study in Canada that evaluated long-term visual outcomes and complications. The results showed that iris-claw Artisan IOL is one of the safest and most efficient alternatives for eye implantation with insufficient capsular support [51]. Previous studies mentioned in this article have also confirmed these findings.

Overall, researchers propose that refractive correction of childhood aphakia is one of the more complicated management issues. Enough capsular support is not observed in several children for allowing an “in the bag” IOL. Therefore, experts in the field have presented alternatives such as contact lenses, surgically fixed IOLs, and spectacles for refractive correction. Though they introduced numerous approaches for IOL fixation, these procedures have not been significantly considered in children. Despite the high attraction of the iris-fixated Artisan aphakic IOL, experts express significant concerns about the IOL de-elevation and corneal ECL rate. Some studies have shown that the use of IFIOLs in children is arguable, and its wide adoption is improbable [11]. To achieve the best results, we must resolve multiple problems with long-term therapeutic options and follow-up [52].

Despite the correlations between anterior Artisan IOLs and side effects, this paper's research showed positive visual outcomes. When Artisan IOLs were fixed behind the pupil, the results were the same as when fixed in front of the pupil or on the sclera. Previous studies have demonstrated VA stability or improved lens subluxation in patients treated with the Artisan IOL placement procedure. We suggest that future research should examine the long-term stability and effectiveness of visual outcomes to evaluate how durable the visual enhancement delivered by the Artisan IOL is. In addition, it is advisable to periodically assess the refractive status of children who have received Artisan IOLs to determine if any changes occur and to evaluate the necessity for further interventions, such as refractive correction. It is also important to examine the occurrence and types of complications associated with Artisan IOL implantation in children, including elevated IOP, lens dislocation, and loss of endothelial cells.

## Conclusions

This comprehensive review showed that it is possible to place, replace, and exchange the Artisan IOL with insignificant surgical trauma. Hence, it was introduced as one of the acceptable therapeutic modalities to correct the developmental refractive changes of the growing aphakic eyes. However, due to probable long-term consequences, including ECL, there are some worries. On the other hand, uncertainties about the long-term safety of each therapeutic alternative for pediatric aphakia are not resolved. Finally, treating pediatric aphakia with Artisan IOL would be seriously considered for visual rehabilitation.
